# Classification Algorithm-Based fMRI Images for Evaluating the Effect of Yishen Tiaodu Acupuncture on the Recovery Period of Cerebral Infarction

**DOI:** 10.1155/2022/3592145

**Published:** 2022-05-25

**Authors:** Zhuo Feng, Miaomiao Hu, Wei Yuan, Xiaojun Zhao, Jiazhi Zeng, Kaibin Zhou

**Affiliations:** ^1^Department of Acupuncture, The First Affiliated Hospital of Guangxi University of Chinese Medicine, Nanning 530023, Guangxi, China; ^2^Department of Sports, Guangxi Medical University, Nanning 530021, Guangxi, China; ^3^Graduate School, Guangxi University of Chinese Medicine, Nanning 530200, Guangxi, China; ^4^Department of Rehabilitation, The Second Affiliated Hospital of Guangxi Medical University, Nanning 530007, Guangxi, China

## Abstract

This study aimed to explore the application value of multifeature fusion classification algorithm based on deep learning and Yishen Tiaodu acupuncture in the diagnosis and treatment of patients with cerebral infarction in convalescence. *Methods*. 62 patients with cerebral infarction were randomly classified into the experimental group and the control group, with 31 patients in each group. All patients received the functional magnetic resonance imaging (fMRI) examination. The image processing method was the multifeature fusion classification algorithm based on deep learning. DICE coefficient, accuracy, and sensitivity were used to evaluate the image processing performance of traditional and new algorithms. Patients in the experimental group were treated with Yishen Tiaodu acupuncture, while patients in the control group were treated with ordinary acupuncture. The evaluation of the cyberchondria severity scale (CSS) and the activities of daily living (ADL) was performed at enrollment, 15 days after treatment, 28 days after treatment, and 1 month after treatment. The results showed that the quality of fMRI images processed by multifeature fusion classification algorithm based on deep learning was signally improved. The clinical efficacy of the traditional Chinese medicine (TCM) syndrome score (86.7% vs. 60.9%) and neurological impairment score (83.4% vs. 53.5%) in the experimental group were remarkably higher compared with the control group (*P* < 0.05). After treatment, the TCM syndrome score of the experimental group was markedly lower than that of the control group, while the ADL score was higher (*P* < 0.05). *Conclusion*. The performance of multifeature fusion classification algorithm based on deep learning in fMRI image processing of patients with cerebral infarction is better than that of traditional algorithms. Yishen Tiaodu acupuncture has a good therapeutic effect on the recovery of motor and neurological function in patients with cerebral infarction at convalescence.

## 1. Introduction

Cerebral infarction is ischemic stroke, which is defined as cerebral ischemia and hypoxic necrosis caused by blood circulation disorder in the brain, and the corresponding neurological impairment [1]. The disease is also easy to relapse. The recurrence rate of cerebral infarction in China is as high as 40%. It is one of the most common cerebrovascular diseases in the elderly in China [2–4]. With the continuous progress of medical technology, more and more patients' lives have been saved [5]. However, the vast majority of patients after surgical treatment are biased disorders, aphasia and other disabilities, which have a great effect on the physical and mental health of patients [6]. At present, the treatment of dysfunction and complications in patients with cerebral infarction by Western medicine is still limited, and there is still a lack of specific treatment measures in the world [7]. Traditional Chinese medicine (TCM) has had remarkable superiority in the treatment of cerebral infarction. In the treatment of TCM, cerebral infarction belongs to the category of stroke. In the acute convalescence period of cerebral infarction, effective treatment can effectively shorten the treatment time of patients, reduce dysfunction, and help patients achieve functional self-care as soon as possible [8, 9]. Acupuncture is a common and effective method to treat cerebral infarction in TCM clinically [10]. TCM believes that the brain dominates the mind and the brain marrow is its material basis. The brain marrow is composed of the kidney-YANG and kidney-YIN. It is up along with the governor vessel and eventually into the brain. It can be seen that kidney, governor vessel, and brain are closely related [11].

The main content of postoperative motor and functional repair in patients with cerebral infarction is nerve repair. The mechanism of nerve repair is very complex. Functional imaging is the main tool to help people understand the repair mechanism after brain injury. The advantages of noninvasive brain function research in living tissues have been widely used by researchers of neurological function in China and abroad [12, 13]. Reviewing previous studies, it is found that most of the relevant studies focus on the research at a single time point, namely, horizontal research. There are few longitudinal studies, that is, to observe the repair process of brain tissue in patients with cerebral infarction in the acute phase and recovery phase. Therefore, it is impossible to understand the mechanism of brain functional reorganization compensation from the perspective of dynamic change [14].

Computer and Internet technologies have gradually penetrated into various fields. It is also applied in the field of auxiliary medical diagnosis [15]. At present, the research on multifeature fusion classification of medical images mainly focuses on modular feature fusion. Therefore, the traditional multifeature fusion classification method cannot obtain excellent processing results. Moreover, improper connection in each method will cause poor fusion results. Therefore, how to solve the disadvantages of traditional image processing modularization has become the focus of research [16]. Multi-feature fusion algorithm is one of the most popular algorithms in recent years. It can extract features directly from original images, without modularization processing. It can greatly improve the fusion effect and speed. However, there are relatively few studies on its clinical adoption, so further research is required.

In this study, a new multifeature fusion classification algorithm based on deep learning is designed and used to process fMRI images of patients with cerebral infarction. On this basis, the therapeutic effect of Yishen Tiaodu acupuncture on cerebral infarction recovery was analyzed. In order to provide reference and basis for clinical research.

## 2. Research Materials and Methods

### 2.1. Research Objects

Sixty-two patients with cerebral infarction in the hospital from June 2019 to October 2020 were selected as subjects and they were randomly divided into experimental group and control group (each with 31 patients). The standards of *The Chinese Society of Traditional Chinese Medicine* issued by the *China Association of Chinese Medicine* in 2010 were adopted for the diagnosis of TCM symptoms in patients with cerebral infarction. *The Clinical Diagnosis and Treatment Guidelines Neurology Volume* published by the *China Association of Chinese Medicine* in 2006 were adopted for the diagnosis of western medicine. This study had been approved by medical ethics committee of the hospital, and all the patients signed the informed consent.

Inclusion criteria were as follows: (1) Patients who met the above diagnostic criteria of TCM and Western medicine and belonged to the recovery period of cerebral infarction (the incidence was greater than 2 weeks and less than 6 months). (2) Stable condition. Unconscious disorder. Vital signs are stable. (3) Patients without previous history of fainting. (4) Clinical basic medication consistent. (5) Patients were fully informed, voluntary cooperation and family consent. Exclusion criteria were as follows: (1) Failure to meet the above diagnostic criteria and inclusion criteria. (2) Patients with acupuncture contraindications. (3) Patients with mental disorders and intellectual disabilities and unable to lie in peace. (4) Long-term drinking and smoking of patients. Patients with previous history of drug abuse. (5) Patients cannot cooperate with the tester.

### 2.2. fMRI Examination Method

Equipment and imaging parameters: MRI data acquisition used a 3.0T HD-X magnetic resonance scanner and head eight-channel phased array coil. The whole brain 3D high-resolution T1WI structural images and fMRI scans were performed on all participants. The scan sequence is shown in Table 1.

### 2.3. Data Processing

The multifeature fusion classification algorithm based on deep learning is used to process the data. The multifeature fusion classification algorithm based on deep learning mainly includes convolution layer, pooling layer, full connection layer, and SoftMax classification layer. (1) shows the calculation method of the convolution process.

(1) $$\begin{array}{c} x_{j}^{l}=f\left(\sum_{i\in M_{j}}x_{j}^{l-1}•K_{ij}^{l}+b_{j}^{l}\right), \end{array}$$

*l* is the number of layers, *K* is the convolution kernel, *x*_*j*_^*l*−1^ is the feature map of the output of the previous layer, *K*_*ij*_^*l*^ is the convolution kernel weight, *b* is the partial value, and *f*(•) is the activation function. Convolution operations have full convolution, same convolution, and valid convolution three modes. Equations (2)–(4) show the specific definition.

(a) Full convolution
  (2) $$\begin{array}{c} \left\{\begin{array}{c} y=\text{conv}\left(x,w,{}^{\prime }\text{full}{}^{\prime }\right)=\left(y\left(1\right),\ldots ,y\left(t\right),\ldots ,y\left(n+m-1\right)\right)\in R,\\ y\left(t\right)=\sum_{i=1}^{m}x\left(t-i+1\right)\cdot w\left(i\right)t=1,2,\ldots ,n+m-1. \end{array}\right. \end{array}$$
(b) Same convolution
  (3) $$\begin{array}{c} y=\text{conv}\left(x,w,{}^{\prime }\text{same}{}^{\prime }\right)\\ =\text{center}\left(\text{conv}\left(x,w,{}^{\prime }\text{full}{}^{\prime }\right),n\right)\in R. \end{array}$$
(c) Valid convolution
  (4) $$\begin{array}{c} \left\{\begin{array}{c} y=\text{conv}\left(x,w,{}^{\prime }\text{valid}{}^{\prime }\right)=\left(y\left(l\right),\ldots ,y\left(t\right),\ldots ,y\left(n+m-1\right)\right)\in R,\\ y\left(t\right)=\sum_{i=1}^{m}x\left(t+i-1\right)w\left(i\right)t=1,2,\ldots ,n+m-1. \end{array}\right. \end{array}$$

The pooling layer can reduce the possibility of overfitting and improve the fault tolerance of the model. (5) shows the expression of the pooling layer.

(5) $$\begin{array}{c} x_{j}^{l}=f\left(\beta_{j}^{l}\text{down}\left(x_{j}^{l-1}\right)+b_{j}^{l}\right). \end{array}$$

*do*  *wn*(•) is the downsampling function. *β* and *b* are multiplicative bias and additive bias, respectively. There are two common pooling operations in multifeature fusion classification algorithm based on deep learning, mean pooling, and max pooling. Mean pooling is the mean within the filter range as pooling output. Maximum pooling is the maximum within the filter range as pooling output. The specific pattern is shown in Figure 1.

Full connection process: In the multi-feature fusion classification algorithm based on deep learning, the full connection layer is a network node with linear arrangement. The output results of the previous layer are coded as one-dimensional vectors. (6) shows the definition of full connection layer.

(6) $$\begin{array}{c} x^{l}=f\left(w^{l}x^{l-1}+b^{l}\right), \end{array}$$

*w*^*l*^ is the network weight coefficient. *x*^*l*−1^ is the output feature map of the upper layer. *b*^*l*^ is the offset item of the full connection layer.

The SoftMax classification layer is a multiclassifier connected to the full connection layer. It can complete more than two categories of classification tasks and convert multiple outputs to probability values in the (0,1) interval. In logical regression, the training set is *T*={(*x*^(1)^, *y*^(1)^),…, (*x*^(*m*)^, *y*^(*m*)^)}, and Enter sample *x*^*i*^ ∈ *R*^*n*^, *y*^(*i*)^ as sample labels. *y*^(*i*)^ ∈ {0,1}. Then, equation (7) shows how the hypothesis function is expressed.

(7) $$\begin{array}{c} h_{\theta }\left(x\right)=\frac{1}{\left(1+e^{-\theta_{X}^{T}}\right)}. \end{array}$$

Equation (8) shows the minimum cost function value of *J*(*θ*).

(8) $$\begin{array}{c} J\left(\theta \right)=-\frac{1}{m}\left[\sum_{i=1}^{m}y^{\left(i\right)}\text{log}h_{\theta }\left(x^{\left(i\right)}\right)+\left(1-y^{\left(i\right)}\right)\text{log}\left(1-h_{\theta }\left(x^{\left(i\right)}\right)\right)\right]. \end{array}$$

Equation (9) shows the calculation of SoftMax.

(9) $$\begin{array}{c} h_{\left(\theta \right)}\left(x^{\left(i\right)}\right)=\left[\begin{array}{c} p\left(y^{\left(i\right)}=1|x^{\left(i\right)},\theta \right)\\ p\left(y^{\left(i\right)}=2|x^{\left(i\right)},\theta \right)\\ \ldots \\ p\left(y^{\left(i\right)}=k|x^{\left(i\right)},\theta \right) \end{array}\right]\\ =\frac{1}{\sum_{j=1}^{k}e^{\theta_{j}^{T}x^{\left(i\right)}}}\left[\begin{array}{c} e^{\theta_{1}^{T}x^{\left(i\right)}}\\ e^{\theta_{2}^{T}X^{\left(i\right)}}\\ \ldots \\ e^{\theta_{K}^{T}x^{\left(i\right)}} \end{array}\right]. \end{array}$$

Learning on the training sample *T* minimizes the damage function of SoftMax. The minimum loss function is expressed as shown in (10).

(10) $$\begin{array}{c} J\left(\theta \right)=-\frac{1}{m}\\ =\left[\sum_{i=1}^{m}\sum_{j=1}^{k}1\left\{y^{\left(i\right)}=j\right\}\text{log}\frac{e^{\theta_{i}^{T}x^{\left(i\right)}}}{\sum_{i=1}^{k}e^{\theta_{i}^{T}x^{\left(i\right)}}}\right], \end{array}$$

1{*y*^(*i*)^=*j*} represents if *y*=*j*, and the value is 1, otherwise it is 0. The smaller the loss function is, the closer it is to the expected goal.

### 2.4. Evaluation Index of Image Processing Results

The performance of the traditional method and the multifeature fusion classification algorithm based on deep learning is evaluated by DICE coefficient, precision, recall, average symmetric surface distance (ASSD), and the Huffman distance. Equations (11)–(13) show how the DICE coefficient, precision, and sensitivity are expressed.

(11) $$\begin{array}{c} \text{DICE}=\frac{2\text{TP}}{\text{TP}+\text{FP}+\text{FN}}\text{,} \end{array}$$

(12) $$\begin{array}{c} \text{precision}=\frac{\text{TP}}{\text{TP}+\text{FP}}\text{,} \end{array}$$

(13) $$\begin{array}{c} \text{recall}=\frac{\text{TP}}{\text{TP}+\text{FN}}\text{.} \end{array}$$

*DICE* coefficient, accuracy, and sensitivity are used to evaluate the accuracy of classification results by volume overlap. However, because there may be boundary differences in areas with more overlap, the average symmetric surface distance and Hoffman distance are used to measure the difference. The smaller the value of these two indicators is, the higher the precision is. Let *A* be the point on the surface of the lesion label. *B* is the point on the surface of the split result. Equations (14) and (15) show the definition of ASSD.

(14) $$\begin{array}{c} \text{ASD}\left(A,B\right)\frac{\sum_{a\in }A{\text{min}}_{b\in B}d\left(a,b\right)}{\left|A\right|}, \end{array}$$

(15) $$\begin{array}{c} \text{ASSD}\left(A,B\right)=\frac{\text{ASD}\left(A,B\right)+\text{ASD}\left(B,A\right)}{2}. \end{array}$$

Hoffman distance is shown in (16):

(16) $$\begin{array}{c} HD\left(A,B\right)=\text{max}\left\{\underset{a\in A}{\text{max}}{\underset{b\in B}{\min}}^{d\left(a,b\right)}\underset{a\in A}{\max}{\underset{b\text{Î}B}{\min}}^{d\left(a,b\right)}\right\}. \end{array}$$

### 2.5. Treatment Methods

Experimental group: Patients in the experimental group were treated with Yishen Tiaodu acupuncture. Operation method: the acupuncture was performed at Baihui, Fengfu, Dazhui, Mingmen, Shenshu, and Taixi. Methods: the even reinforcing-reducing method was adopted at Baihui, Fengfu, and Dazhui, while the twisting and reinforcing method was at Mingmen, Shenyu, and Taixi. The needle was removed 30 minutes later. The acupuncture was performed once a day, with the 6 times as a course of treatment. There was a 1-day interval for every 2 courses of treatment, with a total of 4 courses.

Control group: patients in the control group were treated with ordinary acupuncture. Operation method: the acupuncture was performed at Hegu, Quchi, Zusanli, and Kunlun with the even reinforcing-reducing method. The needle was removed 30 minutes later. The acupuncture was performed once a day, with the 6 times as a course of treatment. There was a 1-day interval for every 2 courses of treatment, with a total of 4 courses.

### 2.6. Observation Indicators

During the treatment, TCM symptom score, clinical neurological deficit score (CSS), and activities of daily living (ADL) ability scale were used to evaluate the efficacy by Barthel score. The observation time points were: inclusion, treatment (15 days of treatment), end of treatment (28 days of treatment), follow-up (1 month after treatment).

### 2.7. Statistical Methods

Statistical analysis of all data was completed by SPSS11.0. Measurement data were expressed as mean ± standard deviation (x(−) ±*s*). *T* test was used to test the significance of patient data before and after surgery. Counting information is expressed in actual numbers and percentages (%). Significance was tested by X^2^ test. *P* < 0.05 was considered statistically significant.

## 3. Results

### 3.1. General Information of Patients

The basic data of the two groups of patients are shown in Table 2 and Figure 2. The analysis of Table 2 shows that the experimental group had 16 male patients, 15 female patients, with an average age of 63.8 ± 6.3 years. The average course of disease was 6.23 ± 1.38 months. There were 13 male patients and 19 female patients in the control group, with an average age of 64.2 ± 5.5 years. The average course of disease was 6.76 ± 1.43 months. The distribution of educational level of the two groups of patients is shown in Figure 2. The analysis of Figure 2 shows that the experimental group of patients with illiteracy in 5 cases, 13 cases of primary school, and junior high school and above in 13 cases. In the control group, 6 patients were illiterate, 11 patients were in primary school, and junior high school and above in 14 cases. There was no significant difference in the basic information such as age, gender, and educational level between the two groups.

### 3.2. Image Display of Typical Diseases

The typical case image processed by the traditional method and the multi-feature fusion classification algorithm based on deep learning is shown in Figure 3. Analysis of Figure 3 revealed that compared with the images obtained by the traditional fMRI data processing algorithm, the images processed by the multi-feature fusion classification algorithm based on deep learning were clearer and the lesions were more prominent. Image quality had been significantly improved.

### 3.3. Image Processing Effect Evaluation

The comparison results of image processing effect between traditional algorithm and multi-feature fusion classification algorithm based on deep learning are shown in Figure 4. The analysis of Figure 4 showed that the traditional algorithm ASSD mean, DICE mean, HD mean, accuracy mean, and sensitivity mean are 5.22, 0.68, 42.31, 0.7, and 0.76, respectively. The mean values of ASSD, DICE, HD, accuracy, and sensitivity of multi-feature fusion classification algorithm based on deep learning are 1.33, 0.84, 22.66, 0.83, and 0.83, respectively. The difference between the indicators of the two methods was statistically significant, *P* < 0.05.

### 3.4. Comparison of Clinical Efficacy of TCM Symptom Scores between the Two Groups of Patients

The clinical efficacy of TCM symptom scores in the two groups is shown in Table 3. According to the analysis of the experimental group, 2 cases were cured, 7 cases were markedly effective, 18 cases were effective, and 4 cases were ineffective, the effective rate was 87.1%. In the control group, 2 cases were cured, 4 cases were markedly effective, 11 cases were effective, and 14 cases were ineffective. The effective rate was 54.8%. The difference in the effective rate between the two groups was statistically significant, *P* < 0.05.

### 3.5. Comparison of Clinical Efficacy of Neurological Deficit Score between the Two Groups of Patients

The clinical efficacy of neurological deficit scores in the two groups is compared as shown in Table 4. Table 4 shows that in the experimental group, 4 cases were cured, 5 cases were markedly effective, 17 cases were effective, and 5 cases were ineffective. The effective rate was 83.8%. The control group 4 cases were cured, 2 cases markedly effective, 12 cases were effective, and 13 cases were ineffective. The effective rate was 58.1%. The difference in the effective rate between the two groups was statistically significant, *P* < 0.05.

### 3.6. Comparison of TCM Symptom Scores

The comparison of TCM symptom scores between the two groups before and after treatment is shown in Figure 5. Analysis of Figure 5 showed that the TCM symptom score of the experimental group before treatment was 17.22 ± 3.65, and the TCM symptom score after treatment was 9.11 ± 4.63. The TCM symptom score of the control group was 17.83 ± 3.67 before treatment and 10.39 ± 4.89 after treatment. The TCM symptom scores of the two groups after treatment were significantly lower than those before treatment, *P* < 0.05. The decrease in the experimental group was higher than that in the control group, *P* < 0.05.

### 3.7. Comparison of Neurological Deficit Scores between the Two Groups of Patients

The comparison of neurological deficit scores between the two groups before and after treatment is shown in Figure 6. Analysis of Figure 6 revealed that the neurological deficit score of the experimental group before treatment was 17.35 ± 3.84. The neurological deficit score after treatment was 9.36 ± 4.73. The neurological deficit score of the control group before treatment was 17.91 ± 3.76. The neurological deficit score after treatment was 10.41 ± 4.65. The neurological deficit scores of the two groups after treatment were significantly lower than those before treatment, *P* < 0.05. The decrease in the experimental group was higher than that in the control group, *P* < 0.05.

### 3.8. Comparison of the ADL Scale Scores of Patients between the Two Groups

Figure 7 shows the comparison of the ADL scores between the two groups before and after treatment. Analysis of Figure 7 showed that the experimental group before treatment activities of daily living (ADL) scale score was 32.46 ± 13.36. The score of activity of daily living (ADL) was 67.88 ± 14.01 after treatment. The score of ADL scale in the control group before treatment was 38.36 ± 12.83. The activity of daily living (ADL) score was 67.63 ± 14.01 after treatment. After treatment, the ADL scores of the two groups were significantly higher than those before treatment (*P* < 0.05). The increase in the experimental group was significantly greater than that in the control group, *P* < 0.05.

## 4. Discussion

Cerebral infarction is a common clinical neurological disease. In China, cerebrovascular disease ranks second in the cause of death after malignant tumors. Cerebral infarction is the leading cause of disability [17]. In recent years, with the continuous progress of modern diagnosis and treatment technology, the rescue rate of acute cerebral infarction has been increasing. Reduced the mortality rate, relatively increased disability rate. It affects the quality of patients' family and social life. It is estimated that 70% of survivors have varying degrees of dysfunction. Therefore, the recovery of cerebral infarction and postoperative function of patients is the focus of current research in the field of cerebrovascular diseases. A large number of clinical data show that the recovery period of cerebral infarction is the best time for functional recovery of patients with cerebral infarction. Therefore, the current research subjects on the postoperative functional recovery of patients with cerebral infarction are mostly patients with cerebral infarction recovery [18].

At present, the existing western medicine technology for the recovery of cerebral infarction is no effective and exact unique method. TCM acupuncture has a long history and unique advantages in the recovery treatment of cerebral infarction patients. In TCM, cerebral infarction belongs to the category of stroke [19]. TCM believes that the situation of liver wind and phlegm fire in patients with stroke recovery has recovered. The illusion has gradually emerged. However, wind, fire, phlegm, and blood stasis still stagnate meridians. Qi and blood run poorly. Therefore, patients have symptoms of limb paralysis, language disadvantage, restless, limb swelling, dementia, and other symptoms. This disease in the pathogenesis is the virtual standard real, the upper and lower virtual. The virtual real heavy in this virtual, this virtual is kidney essence deficiency. Blood deficiency is cerebral vein malnutrition. The marrow sea emptiness, causes the body function activity barrier [20]. Therefore, the treatment principle of this period is tonifying kidney, promoting blood circulation, and removing blood stasis. Kidney regulating acupuncture can play such a role. And a large number of clinical data show that acupuncture for stroke recovery in patients with motor and neurological recovery has a better effect [21]. In this work, the patients with cerebral infarction were treated with the Yishen Tiaodu acupuncture. The selection of point was scientific and reasonable. The main basis was as follows. The acupuncture to the governor vessel of Baihui, Fengfu, Dazhui, and Mingmen could adjust the governor vessel, awaken the brain, and mobilize the essence of the viscera. Taixi was the original point of kidney meridian, and Shenshu and Mingmen were the points of kidney meridian qi infusion. The acupuncture at the three points could nourish the kidney and essence to the brain, thus nourishing the primordial spirit. All points could stimulate qi, adjust the whole body viscera qi and blood operation, nourish the brain, and awaken the brain.

The fMRI technology not only makes early, accurate, and rapid diagnosis of cerebral infarction possible. It can also provide imaging data for metabolic changes, treatment, and prognosis in patients with cerebral infarction [22]. Compared with other brain function examination techniques, IMRI has the characteristics of non-invasive, high spatial resolution, flexibility, and strong interdisciplinary [23]. In summary, fMRI has a unique advantage in the diagnosis and treatment of cerebral infarction patients in recovery period. In recent years, computer and Internet technology continues to progress and development, which gradually penetrated into all aspects of people's lives. It has also been greatly developed in the field of medical image processing. The most important part of medical image processing is feature extraction. The multi-feature fusion algorithm is the most commonly used feature extraction algorithm [24]. However, with the continuous development of deep learning algorithm, it shows better performance in feature extraction than traditional multi-feature fusion algorithm. It has the tendency to replace the traditional algorithm gradually [25].

In this study, depth-based multi-feature fusion algorithm was used to process fMRI images of patients with cerebral infarction in recovery period. On this basis, the curative effect of Yishen Tiaodu acupuncture on patients with cerebral infarction in recovery period was discussed. It is found that the performance of multi-feature fusion algorithm based on depth is better than that of the traditional algorithm in fMRI image processing of patients with cerebral infarction recovery. Moreover, the therapeutic effect of Yishen Tiaodu acupuncture on patients with cerebral infarction recovery was significantly higher than that of ordinary acupuncture.

## 5. Conclusion

In this study, the fMRI images of patients with convalescent cerebral infarction were processed by multifeature fusion algorithm based on depth. On this basis, the curative effect of Yishen Tiaodu acupuncture on patients with cerebral infarction in the recovery period was discussed. It is found that the performance of multifeature fusion algorithm based on depth was better than that of the traditional algorithm in fMRI image processing of patients with cerebral infarction recovery. The therapeutic effect of Yishen Tiaodu acupuncture on patients with cerebral infarction at recovery stage was significantly higher than that of ordinary acupuncture. Due to the limited sample and space, this study is not comprehensive and in-depth, so the sample will be further expanded and studied in the future study and work.

## Figures and Tables

**Figure 1:** Pooling diagram. (a) Maximum pooling; (b) mean pooling.

**Figure 2:** Educational level distribution of patients in the two groups.

**Figure 3:** Typical case image.

**Figure 4:** Comparison of image processing effects between the traditional algorithm and multi-feature fusion classification algorithm based on deep learning. *∗*Compared with traditional method, *P* < 0.05.

**Figure 5:** Comparison of TCM symptom scores between the two groups before and after treatment. ^*∗*^Compared with before treatment, *P* < 0.05.

**Figure 6:** Comparison of neurological deficit scores between the two groups. ^*∗*^Compared with before treatment, *P* < 0.05.

**Figure 7:** Comparison of ADL scores between the two groups of patients. ^*∗*^Compared with before treatment, *P* < 0.05.

**Table 1:** Image acquisition scanning parameters.

Scanning parameters	The fMRI imaging technology
Repeat time TR (ms)	1800
Echo timeTE (ms)	35
Flip angle FA (°)	90
Lamination thickness (mm)	3.25
Visual field FOV (mm^2^)	256 × 256
Matrix	256 × 256
Tier number	40
Interval (mm)	1
Acquisition phase	180
Scanning time (s)	440

**Table 2:** Comparison of gender, age, and course of disease between the two groups.

Group	Number of samples	Sexuality		Age (years)	Course of disease (months)
		Male	Female		
Experimental group	31	16	15	63.8 ± 6.3	6.23 ± 1.38
Control group	31	12	19	64.2 ± 5.5	6.76 ± 1.43

**Table 3:** Comparison of TCM symptom score and clinical efficacy between the two groups.

Group	The number of cases	Heal	Effectual	Have the effect	Nullification	Effective rate
Experimental group	31	2	7^*∗*^	18^*∗*^	4^*∗*^	87.1%^*∗*^
Control group	31	2	4	11	14	54.8%

^*∗*^Compared with the control group, *P* < 0.05.

**Table 4:** Comparison of clinical efficacy of neurological deficit scores between the two groups.

Group	The number of cases	Heal	Effectual	Have the effect	Nullification	Effective rate
Experimental group	31	4	5^*∗*^	17^*∗*^	5^*∗*^	83.8%^*∗*^
Control group	31	4	2	12	13	58.1%

Compared with the control group ^*∗*^*P* < 0.05.

## Data Availability

The data used to support the findings of this study are available from the corresponding author upon request.
